RETRACTED

# Molecular isoforms of high-mobility group box 1 are mechanistic biomarkers for epilepsy

**DOI:** 10.1172/JCI92001

**Published:** 2017-05-15

**Authors:** Lauren Elizabeth Walker, Federica Frigerio, Teresa Ravizza, Emanuele Ricci, Karen Tse, Rosalind E. Jenkins, Graeme John Sills, Andrea Jorgensen, Luca Porcu, Thimmasettappa Thippeswamy, Tiina Alapirtti, Jukka Peltola, Martin J. Brodie, Brian Kevin Park, Anthony Guy Marson, Daniel James Antoine, Annamaria Vezzani, Munir Pirmohamed

**Affiliations:** 1 Department of Molecular and Clinical Pharmacology, University of Liverpool, Liverpool, United Kingdom.; 2 Department of Neuroscience and; 3 Department of Oncology, IRCCS-Istituto di Ricerche Farmacologiche Mario Negri, Milano, Italy.; 4 Department of Biomedical Sciences, College of Veterinary Medicine, Iowa State University, Ames, Iowa, USA.; 5 Department of Neurology and Rehabilitation, Tampere University Hospital, Tampere, Finland.; 6 Epilepsy Unit, Western Infirmary, Glasgow, United Kingdom.

## Abstract

Approximately 30% of epilepsy patients do not respond to antiepileptic drugs, representing an unmet medical need. There is evidence that neuroinflammation plays a pathogenic role in drug-resistant epilepsy. The high-mobility group box 1 (HMGB1)/TLR4 axis is a key initiator of neuroinflammation following epileptogenic injuries, and its activation contributes to seizure generation in animal models. However, further work is required to understand the role of HMGB1 and its isoforms in epileptogenesis and drug resistance. Using a combination of animal models and sera from clinically well-characterized patients, we have demonstrated that there are dynamic changes in HMGB1 isoforms in the brain and blood of animals undergoing epileptogenesis. The pathologic disulfide HMGB1 isoform progressively increased in blood before epilepsy onset and prospectively identified animals that developed the disease. Consistent with animal data, we observed early expression of disulfide HMGB1 in patients with newly diagnosed epilepsy, and its persistence was associated with subsequent seizures. In contrast with patients with well-controlled epilepsy, patients with chronic, drug-refractory epilepsy persistently expressed the acetylated, disulfide HMGB1 isoforms. Moreover, treatment of animals with antiinflammatory drugs during epileptogenesis prevented both disease progression and blood increase in HMGB1 isoforms. Our data suggest that HMGB1 isoforms are mechanistic biomarkers for epileptogenesis and drug-resistant epilepsy in humans, necessitating evaluation in larger-scale prospective studies.

## Introduction

Epileptogenesis is a dynamic process of molecular, cellular, and functional reorganization following precipitating events that leads to brain pathology capable of generating spontaneous seizures (1). Currently used antiepileptic drugs (AEDs) merely provide symptomatic control of seizures, and around 30% of patients have epilepsy that is refractory to AEDs (2). The development of effective therapies to treat or prevent epileptogenesis and drug resistance remains an urgent unmet clinical need. Clinical trial designs for novel therapeutics against epileptogenesis are likely to hinge on discovering noninvasive biomarkers that allow early identification of patients at high risk of developing the disease as well as patients who might preferentially respond to novel treatments.

RETRACTED

Neuroinflammation in seizure-prone brain regions is a common feature of various forms of drug-resistant, focal-onset symptomatic epilepsies in humans and contributes to mechanisms of seizure generation in animal models (3). Sterile neuroinflammation is a complex phenomenon involving the activation of the innate immune system by damage-associated molecular patterns (DAMPs). DAMPs are released by cells undergoing stressful or deadly events to alert the microenvironment to activate homeostatic mechanisms of tissue repair, but if DAMPs persist in tissue, they may induce cell dysfunction or damage (4). High-mobility group box 1 (HMGB1), a prototypical member of the DAMP family, is a known mediator of sterile neuroinflammation evoked by epileptogenic injuries (4, 5). HMGB1 is a highly conserved nonhistone nuclear protein expressed by most eukaryotic cells, where it binds to chromatin (6) and regulates gene transcription (7). HMGB1 has several isoforms, each of which has distinct physiological and pathological functions. Nonacetylated HMGB1 is released passively from necrotic cells (7), while acetylation of key lysine residues in HMGB1 indicates active release during inflammation, a step that requires nucleus-to-cytoplasm translocation (6, 8). Furthermore, the redox state of the protein determines its receptor interactions: under basal conditions, HMGB1 is predominantly fully reduced inside the cell, but can be oxidized by reactive oxygen species upon translocation to the cytoplasm or after its extracellular release. Redox modification of 3 key cysteine residues, C23, C45, and C106, determines the functional activity of HMGB1. In particular, disulfide HMGB1, containing an intramolecular disulfide bond between C23 and C45 and a reduced C106 (9), specifically binds and signals via the TLR4/MD-2 complex to induce cytokine release in macrophages (10), microglia, and astrocytes (5, 11, 12). Reduced HMGB1, in which all 3 cysteines are reduced, forms a heterocomplex with the C-X-C motif chemokine 12 (CXCL12) and binds CXCR4 to initiate chemotaxis (13). HMGB1 that is terminally oxidized to contain sulfonyl groups on all cysteines (sulfonyl HMGB1) does not affect cell migration or cytokine induction (14). The disulfide and reduced isoforms have mutually exclusive functions. HMGB1 also activates receptor for advanced glycation end products (RAGE), but the binding efficiency of each isoform for RAGE is still unresolved.

RETRACTED

We have shown that total HMGB1 and its nucleus-to-cytoplasm translocation increase in neurons and glia in human drug-resistant epileptic foci (5, 12) and the corresponding animal models (5) and that disulfide HMGB1 is the isoform that promotes seizures and cell loss (5, 15, 16). Furthermore, mice lacking TLR4 or RAGE are intrinsically less susceptible to seizures and less prone to developing epilepsy (5, 15), suggesting that HMGB1 is implicated in epileptogenesis and that therefore, its targeting may have therapeutic utility. However, the role of HMGB1 and its different isoforms in both epileptogenesis and drug resistance, including whether they can be used as noninvasive, mechanistic biomarkers of epileptogenesis and treatment response, is unclear. In order to address this, we have measured total HMGB1 and its acetylated, reduced, and disulfide isoforms before epilepsy onset and during disease development in animal models of acquired epilepsy, correlating brain changes to those in blood, and have undertaken bridging studies in well-defined patients with drug-refractory epilepsy and in newly diagnosed patients.

## Results

### Brain expression and blood levels of HMGB1 in rodent models of epilepsy.

Our first objective was to establish whether a relationship exists between brain and blood levels of HMGB1 during the acute injury and early epileptogenesis following status epilepticus (SE), a brain insult leading to epilepsy in animal models and humans (17, 18). We investigated whether HMGB1 translocates from the nucleus to the cytoplasm during epileptogenesis (Figure 1A), since this step is required for its cellular release, the consequent biological effects (19), and its potential brain-to-blood transfer. Cellular localization of HMGB1 was assessed immunohistochemically in the hippocampus of rats exposed to electrically induced SE, a well-characterized model of epilepsy (20, 21), and these hippocampi were compared with sham controls (see Supplemental Methods; supplemental material available online with this article; https://doi.org/10.1172/JCI92001DS1). In control tissue, HMGB1 was expressed in nuclei of neurons and glia (Figure 1A and Supplemental Figure 1). From 3 hours until 4 days after SE, a time window preceding the onset of epilepsy in this model, as shown by the lack of EEG and motor seizures in rats under continuous video-EEG recording (spontaneous seizures arise at 8.4 ± 1.8 days, see below), HMGB1 staining showed a progressive increase in GFAP-positive astrocytes (Figure 1A and Supplemental Figure 2). Notably, in all SE-exposed rats, HMGB1 staining was observed in the cytoplasm of glial cells, including activated OX-42–positive microglia, and in endothelial barrier antigen–positive (EBA-positive) endothelial cells of the blood brain barrier (BBB) (Figure 1A) and was detectable in the cytoplasm of neurons in 30% of animals (Supplemental Figure 1). These data show that HMGB1 translocates from nucleus to cytoplasm before the onset of spontaneous seizures, therefore demonstrating that brain changes of HMGB1 are not solely a consequence of ongoing seizure activity.

RETRACTED

Liquid chromatography–tandem mass spectrometry (LC/MS-MS) analysis of HMGB1 isoforms was subsequently performed in both hippocampus and blood in a different cohort of rats that were sacrificed at representative time points after SE, as informed by the immunohistochemical analysis. The proteolytic digestions of HMGB1 required for LC/MS-MS analysis generates peptide fragments that either contain the acetylation sites or the redox sensitive sequence (Supplemental Figure 3). HMGB1 isoforms in serum have been determined by a patented absolute quantification method (22, 23), which has been extensively validated to bioanalytical guidelines set out by the biomarker consortium funded by the Safer and Faster Evidence-Based Translation Innovative Medicines Initiative (SAFE-T IMI) (http://www.imi-safe-t.eu/). Since a method for absolute quantification of HMGB1 isoforms has not been validated for brain tissue as yet, HMGB1 isoforms in brain are expressed as fold change of respective basal values. The results depict acetylated HMGB1 separately from the reduced and disulfide isoforms. Since reduced and disulfide HMGB1 are mutually exclusive isoforms, their amounts account for total HMGB1 levels.

We determined whether an association exists between brain and blood HMGB1 isoforms (Figure 1B and dot plots in Supplemental Figure 4). In brain lysate from hippocampal tissue, the acetylated isoform (indicator of active release) progressively increased between 3 hours and 4 days after SE, i.e., during a time frame preceding the onset of spontaneous seizures. The redox state of HMGB1 also changed during epileptogenesis: at 3 hours after SE, only reduced HMGB1 was formed (3-fold increase over sham value, not statistically significant). However, between 6 hours and 4 days, disulfide HMGB1 was also generated together with reduced HMGB1. In the blood of the same animals, the acetylated and disulfide isoforms increased with a delay of at least 6 hours when compared with brain and before spontaneous seizure onset. The reduced isoform increased in blood concomitantly with brain changes and, as in brain, anticipated the generation of disulfide HMGB1, which appeared in blood at 4 days. Within the first 6 hours from SE induction, circulating HMGB1 was nonacetylated, reflecting its passive release from damaged cells, while at 4 days, the majority of HMGB1 was acetylated, indicating active cellular release. It has previously been shown that the active cellular release of HMGB1 is through a Ca^2+^-dependent secretory lysosome mechanism that, in turn, depends on HMGB1 acetylation (24, 25).

RETRACTED

These blood changes may reflect cerebrospinal fluid–to–blood (CSF-to-blood) transport of HMGB1, which is initially (within the first 3 hours) passively released from damaged neurons (5, 26) and possibly also from BBB endothelium (27, 28). In particular, at 3 hours after SE, nonacetylated and reduced HMGB1 in blood overshot the brain changes by about 2-fold, suggesting an additional cellular source of HMGB1 other than the brain parenchyma, such as the brain endothelium. In accordance, endothelial cells showed increased expression of HMGB1 during epileptogenesis (Figure 1A). Further, it has previously been demonstrated that endothelial cells can be damaged by SE (29), suggesting that these cells may serve as a source of HMGB1.

The progressive active release of acetylated HMGB1 may originate mainly from astrocytes, as suggested by both the prominent astrocytic HMGB1 expression and its cytoplasmic translocation by immunohistochemistry (Figure 1A and Supplemental Figure 2).

Notably, the brain changes in both acetylated and disulfide isoforms preceded the respective blood increases, supporting a CSF-to-blood transport. We cannot exclude, however, that leukocytes contribute to blood HMGB1 changes. Both the hypothalamic-pituitary-adrenal (HPA) axis and the vagal nerve can mediate signaling of the inflammatory state in the brain to the blood, and this phenomenon could promote the release of HMGB1 from circulating leukocytes. It should be noted, however, that these brain-to-blood signals usually result in peripheral antiinflammatory (rather than proinflammatory) responses (30).

To exclude model-specific changes, we also measured HMGB1 in blood of adult male C57BL/6J mice exposed to SE induced by systemic kainate (31). As in rats, we found on average a 3-fold increase in reduced HMGB1 between 3 hours and 6 hours after SE, while both the acetylated and disulfide isoforms were unchanged (not shown).

RETRACTED

### HMGB1 as a biomarker in animal models.

To investigate the value of blood HMGB1 in predicting epilepsy development (Figure 2 and Supplemental Figure 5A), we used the electrically induced SE model (also used in Figure 1) in which all rats develop epilepsy to test whether blood HMGB1 levels change before the onset of the spontaneous seizures independently of ongoing seizure activity. We measured blood HMGB1 longitudinally at 3 times after SE that are representative of disease development: 7 days (preceding spontaneous seizure onset), 14 days (early after disease onset), and 4.5 months (chronic epilepsy phase). Using the same model, we also tested the utility of blood HMGB1 for predicting a therapeutic response to antiinflammatory drugs. Rats exposed to electrical SE were randomized in 1 treatment group (*n* = 9) injected with a combination of antiinflammatory drugs during epileptogenesis and 1 placebo group (*n* = 9), which received the corresponding vehicles. Drugs or their vehicles were injected into rats for 1 week starting 1 hour after SE induction (Supplemental Figure 5A and Supplemental Figure 6, A and B) to encompass the epileptogenesis phase preceding disease onset; then treatment was stopped. Rats were video-EEG monitored continuously from the induction of SE until the first spontaneous seizures (i.e., epilepsy onset). Spontaneous seizures were counted for 2 weeks at 2.0 and 4.0 months as the primary outcome measure. Based on our background evidence (5, 15, 20), we used a rational combination of antiinflammatory drugs, anakinra, (the human recombinant IL-1 receptor antagonist, ref. 32; 10 mg/200 μl/rat, i.v.) and BoxA (a fragment of HMGB1 with antagonist activity, ref. 33; 100 μg/200 μl/rat, i.v.) together with ifenprodil (a blocker of the NR2B-containing NMDA receptor [NMDAR], ref. 34; 20 mg/kg, i.p.) (treatment protocol in Methods). This treatment combination was designed to efficiently block the activation of the IL-1R1/TLR4 pathway, a known contributor to seizure mechanisms (4), as well as a key molecular target (the NR2B-NMDAR) that mediates increased neuronal excitability induced by pathway activation (16, 35). In fact, our previous evidence showed that the single blockade of the IL-1R1 axis was not sufficient to prevent TLR4 signaling activation during epileptogenesis (20) and that TLR4 signaling itself contributes to epileptogenesis (15). A group of vehicle-injected rats implanted with electrodes but not exposed to SE was used as a sham control for time-matched blood HMGB1 measurements (*n* = 9).

We found a progressive increase of both total HMGB1 and its acetylated and disulfide isoforms (the latter being undetectable in sham rats) in blood during disease development in vehicle-injected rats; notably, these changes were detected before the onset of the spontaneous seizures (i.e., disease onset), as assessed in rats continuously monitored by video-EEG, and persisted until the chronic phase of spontaneous seizures (Figure 2 and dot plots in Supplemental Figure 7). Before disease onset, acetylated HMGB1 was the predominant isoform (7 days, mean 70% of total HMGB1) reflecting active release. This isoform plateaued early after disease onset (14 days, mean 50%) and increased again in the chronic disease phase (4.5 months, mean 80%). Reduced HMGB1 stably increased around 4-fold throughout the observation period (Figure 2; dot plots in Supplemental Figure 7). The inactive sulfonyl HMGB1 was not detected at any time point.

RETRACTED

The antiinflammatory drug combination significantly attenuated the increase in total HMGB1 and its isoforms during the prodromal phase and abrogated blood HMGB1 changes after disease onset (Figure 2; dot plots in Supplemental Figure 7). Notably, the drug combination also prevented the increase in seizure frequency determined by EEG analysis between 2.0 and 4.5 months after SE in vehicle-injected rats (Figure 3; Supplemental Table 1), thus indicating that the antiinflammatory drugs prevented disease progression. An additional salutary effect of treatment was prevention of body weight loss occurring in SE-exposed rats (Supplemental Figure 5B).

The drug combination did not modify the duration or severity of SE (Supplemental Figure 6, A and B) and the consequent neurodegeneration (Supplemental Figure 8 and Supplemental Methods) or the time of spontaneous seizure onset (SE+vehicle, 8.4 ± 1.8 days; SE+drug, 11.6 ± 1.7 days, *n* = 9 each group). Receiver operating characteristic (ROC) analysis (Table 1) showed that both total HMGB1 and its isoforms reliably differentiated between sham control and epileptic rats (AUC = 1) in the chronic phase of spontaneous seizures, supporting their value as diagnostic biomarkers of active epilepsy. Additionally, total HMGB1 and its isoforms also predicted with high fidelity (AUC = 0.8–1 range) the therapeutic response to antiinflammatory drugs before disease onset and at epilepsy diagnosis.

There was no correlation between the number of chronic seizures in the 2-week recording period preceding blood withdrawal (4.5 months after SE) and the corresponding level of total blood HMGB1 (Supplemental Figure 9A).

Since the changes in blood HMGB1 were detected in rats before the onset of the disease, we continued our investigations to validate the potential role of HMGB1 for predicting epilepsy development. In a subsequent study, we evoked SE by systemic lithium+pilocarpine in preadolescent (P21) rats (Supplemental Figure 5C), since only around 70% of rats develop epilepsy after an average time of 70 days (36–40). In this model, 12 out of 17 rats developed spontaneous seizures after being exposed to SE of similar severity (Supplemental Figure 6C) and duration (26.3 ± 0.5 hours). Blood was drawn longitudinally after SE at 23 days (prodromal phase), 73 days (encompassing the time of disease onset in 70% of rats), and 7.5 months (chronic epilepsy phase) (Supplemental Figure 5C). In the chronic epilepsy phase, we counted spontaneous seizures during 2 weeks of continuous video-EEG monitoring: epileptic rats experienced 3.7 ± 0.5 clinical seizures, while no seizures were observed in nonepileptic rats. Epileptic rats also displayed a significant reduction in the threshold to afterdischarge (ADT) induction (116 ± 38 μA, *n* = 12; *P* < 0.05) as compared with sham controls (220 ± 40 μA, *n* = 7); nonepileptic rats without spontaneous seizures were similar to controls (190 ± 40 μA, *n* = 5). For HMGB1 blood measurement, we randomly selected 5 epileptic rats (4.0 ± 1.3 seizures/2 weeks) and compared them with 5 nonepileptic rats and 7 vehicle-treated sham controls. Only rats who developed epilepsy had increased blood levels of both total HMGB1 and its isoforms; these changes occurred before the onset of the disease and were maintained during disease development (Figure 4A; dot plots in Supplemental Figure 10). Nonepileptic rats were similar to controls at all time points after SE (Figure 4A; dot plots in Supplemental Figure 10). The inactive sulfonyl HMGB1 isoform was not detected under any experimental conditions. Moreover, postmortem brain analysis showed that only epileptic rats displayed increased HMGB1 expression in the hippocampus at 7.5 months with concurrent nucleus-to-cytoplasm translocation in glial cells, while nonepileptic rats were similar to controls (Figure 4B). ROC analysis showed perfect discrimination between epileptic and nonepileptic rats (AUC = 1; Table 2), with both total HMGB1 and its isoforms measured either before the onset of spontaneous seizures (Supplemental Figure 11), at the onset of disease, or in the chronic epilepsy phase (Table 2). The blood changes in HMGB1 did not merely reflect reactive gliosis, since the hippocampal level of myo-inositol, a metabolite reflecting astrocyte activation, was similarly augmented (*P* < 0.05) in all rats either with or without HMGB1 blood increase, as assessed by proton magnetic resonance spectroscopy (^1^H-MRS) 23 days after SE at the time of blood withdrawal (Supplemental Figure 12A). Moreover, the level of gliosis assessed in these rats 7.5 months after SE by postmortem glial fibrillary acidic protein (GFAP) immunostaining was similar in the hippocampus of rats with epilepsy (showing elevated blood HMGB1) or without epilepsy (with no elevation of blood HMGB1) (Supplemental Figure 12B).

RETRACTED

Hippocampal cell loss in CA3 pyramidal cell layer and hilus was detected in epileptic rats (*n* = 5) versus sham controls (not exposed to SE, *n* = 7): number of cells, CA3, sham, 546 ± 54; epileptic, 454.5 ± 13 (*P* < 0.05); hilus, sham, 93.9 ± 7.1; epileptic, 38.9 ± 2.9 (*P* < 0.01). Nonepileptic rats had a pattern and extent of cell loss similar to those in epileptic rats (not shown).

### HMGB1 allows stratification of patients with pharmacoresistant epilepsy.

Because HMGB1 was increased in both brain and blood in rats with active epilepsy and its levels were modulated by therapeutic interventions that reduced seizures, we hypothesized that total HMGB1 and its isoforms may be used as biomarkers for drug resistance in human epilepsy. We examined HMGB1 levels in sera from 65 patients with drug-resistant epilepsy undergoing continuous inpatient video-EEG monitoring, 20 patients with well-controlled epilepsy (diagnosed more than 12 months previously, seizure-free for more than 6 months on AED therapy) included as drug-responsive epilepsy controls, and 74 healthy controls (Supplemental Tables 2–4). Patients with drug-resistant epilepsy expressed significantly higher levels of total HMGB1 (8.70 ± 0.47 ng/ml) than both healthy controls (1.11 ± 0.07 ng/ml, *P* < 0.01) and those with well-controlled epilepsy (1.25 ± 0.15 ng/ml, *P* < 0.01; Figure 5A). Patients with abnormal brain MRI showed significantly higher HMGB1 levels (mean ± SEM, 9.8 ± 0.7 ng/ml, *n* = 35) than those without imaging abnormalities (7.4 ± 0.5 ng/ml, *n* = 30, *P* < 0.01; Supplemental Figure 13). Notably, acetylated HMGB1 was observed in drug-resistant epilepsy patients, but not in controls or drug-responsive patients. Patients with drug-resistant epilepsy could be further stratified on the basis of the presence of the disulfide isoform (Figure 5A). There was no significant association between the presence of disulfide HMGB1 and any of the clinical variables (Supplemental Table 2). Furthermore, there was no correlation between the number of seizures in the preceding month and the level of total HMGB1 in blood (Supplemental Figure 9B).

For the comparison between control values and those obtained from patients that were drug resistant, a total ROC-AUC of 0.99 (*P* = 0.0001) was recorded (Figure 5B). The sensitivity at 95% specificity gave an ROC-AUC of 0.94 (95% CI 0.85–0.98) with a cut-off HMGB1 concentration of 2.3 ng/ml. For the comparison between values from patients with well-controlled epilepsy and those obtained from patients that are drug resistant, a total ROC-AUC of 0.99 (*P* = 0.0001) was recorded (Figure 5B). The sensitivity at 95% specificity gave an ROC-AUC of 0.93 (95% CI 0.85–0.99), which also had a cut-off of HMGB1 concentration of 2.3 ng/ml (for values used to determine ROC).

RETRACTED

### HMGB1 in newly diagnosed epilepsy.

In a pilot study, we examined HMGB1 isoforms in the peripheral blood of 27 patients with newly diagnosed epilepsy. The acetylated and disulfide isoforms of HMGB1 (DS-A) were detectable at diagnosis (i.e., baseline visit) in 25 of 27 patients (median, 2.00 ng/ml; range, 0.0-8.10), with 2 patients falling below the quantifiable limit. There was no significant correlation between the total pretreatment seizure count at diagnosis and the corresponding amount of HMGB1 present in blood (Supplemental Figure 14). Nor was there any significant relationship between the number of days since the last seizure and the total amount of blood HMGB1 present (Supplemental Figure 15).

At the 6-week follow-up visit, 13 of 27 patients were seizure free (median DS-A, 0.8 ng/ml; range, 0.0–7.40). The remaining 14 patients who had experienced subsequent seizures had significantly higher DS-A levels (median DS-A, 3.25 ng/ml; range, 0.0–10.60, *P* = 0.04), with no patients having undetectable levels. Five of the seizure-free patients had undetectable DS-A levels at 6 weeks; 4 of these patients remained seizure free at 6 months, while a further patient was also seizure free, but no sample was available for analysis.

By 6 months, 5 patients were lost to follow-up. Eleven patients were seizure free (median DS-A, 0.0 ng/ml; range, 0.0–8.70); in 7 of the patients, DS-A levels were undetectable. The remaining 11 patients had subsequent seizures, and they had significantly higher DS-A levels (median DS-A, 8.30 ng/ml; range, 0.0–8.90, *P* = 0.02).

An additional 2 patients recruited to the study had their epilepsy diagnosis revised to nonepileptic attack disorder (NEAD). DS-A HMGB1 isoform was absent in these 2 patients. It was not detectable in the sera of healthy human subjects (41) or patients with well-controlled chronic epilepsy who were seizure free (Figure 5A).

## Discussion

Our comprehensive assessment shows that circulating isoforms of HMGB1 may serve as mechanistic biomarkers of epileptogenesis in animal models as well as drug-resistant epilepsy in humans. Electrically induced SE in adult rodents increased nonacetylated and reduced HMGB1 isoforms in blood within hours. This is consistent with passive release of HMGB1 from injured neuronal and endothelial cells (5, 9), which is known to occur in the hippocampus after SE (26, 27). Following a different pilocarpine-induced epileptogenic insult, we also identified an early increase in nonacetylated and reduced HMGB1 in the blood of rats that developed epilepsy, but not in those who did not, despite similar neuronal cell loss. Thus, this evidence suggests that the passive release of HMGB1 following SE not only reflects cell death, but may also be a marker of the overall state of cell stress in neurons, glia, and BBB endothelium induced by the epileptogenic insult.

RETRACTED

At later time points of epileptogenesis, notably before the onset of spontaneous seizures and during disease development in the 2 animal models, both acetylated and disulfide isoforms progressively increased and accounted for the majority of total HMGB1 blood levels. This phenomenon is consistent with active release of HMGB1 from activated glial cells, as supported by immunohistochemistry, and it may therefore reflect either HMGB1 brain-to-blood leakage due to BBB damage (27) or CSF-to-blood diffusion (42), although we cannot exclude a contribution of peripheral leukocytes to HMGB1 blood changes (43). Total HMGB1 and all its isoforms increased in blood before the onset of spontaneous seizures, and these changes persisted only in animals with active epilepsy. Importantly, blood HMGB1 predicted which animal would develop the disease with high fidelity (AUC = 1). On that basis, it is possible that blood HMGB1 might identify patients with the highest risk of developing spontaneous seizures early after a potentially epileptogenic injury. This hypothesis can be tested in prospective human clinical studies, such as in poststroke or posttraumatic epilepsy, by examining the prognostic value of total HMGB1 and its isoforms before the first presentation of seizures.

While reduced HMGB1 has chemoattractant properties for macrophage/microglia (6, 9), disulfide HMGB1 induces proinflammatory cytokine release from immune cells by activating TLR4 (6, 9) and contributes to hyperexcitability and seizures in animal models by modulating Ca^2+^ permeability of NR2B-NMDAR (5, 15, 16). Additionally, TLR4 has been implicated in epileptogenesis (15). Therefore, the release of disulfide HMGB1 in the brain following SE may contribute to epileptogenesis and the consequent onset of spontaneous seizures (personal communications, Vezzani). Accordingly, disulfide HMGB1 was generated in the rat brain before the onset of spontaneous seizures. Moreover, only rats who developed epilepsy, but not those without disease or controls, expressed this isoform in blood. The persistence of the pathological disulfide isoform in animals who developed epilepsy probably reflects inefficient resolution of neuroinflammation (36, 44).

RETRACTED

In order to determine the relevance of our findings in animals, we undertook bridging studies in patients with drug-resistant and newly diagnosed epilepsy. Patients with longstanding, drug-resistant epilepsy had significantly (*P* < 0.01) higher total HMGB1 levels in blood compared with patients with well-controlled epilepsy or healthy controls. Only patients with drug resistance expressed the acetylated, actively secreted form of HMGB1. This is consistent with our previous study that showed cytoplasmic translocation of HMGB1 in neurons and glia in human brain tissue taken at epilepsy surgery from drug-resistant patients (5, 12). Notably, blood HMGB1 levels were higher in patients with MRI abnormalities known to be associated with a greater risk of developing drug resistance (45), possibly reflecting more extensive reactive gliosis due to structural damage. Furthermore, a subset of drug-resistant patients expressed disulfide HMGB1, but there was no association between disulfide HMGB1 and any clinical parameter in our patients. It is possible that this particular isoform may allow identification of patients with pathological neuroinflammation analogous to that seen in the P21 rat model (36) and that these patients may be the most amenable to immunomodulatory/antiinflammatory therapies.

Consistent with our findings in animal models, a pilot study in newly diagnosed patients revealed the presence of pathological HMGB1 isoforms not normally seen in the sera of healthy individuals or patients with longstanding, well-controlled epilepsy. Persistent elevation of these pathological isoforms 6 weeks following diagnosis was associated with subsequent seizures, whereas disappearance of this isoform, despite elevated total HMGB1 levels, appeared to indicate a reduced likelihood of subsequent seizures. Our data suggest that certain HMGB1 isoforms that are elevated early in the disease course may be useful prognostic and predictive biomarkers of ongoing seizure activity despite AED therapy. A limitation of our findings was the small number of patients studied. Thus, a prospective, longitudinal study in newly diagnosed patients with epilepsy is required to further investigate this aspect.

Our data in animals and humans indicate that the changes in blood HMGB1 are not solely reflecting ongoing seizure activity or reactive gliosis. In both of the animal models of epilepsy, such changes occurred before the onset of spontaneous seizures. Secondly, HMGB1 blood levels did not correlate with the number of seizures experienced by the animals or by patients with epilepsy (Supplemental Figures 9 and 14). Finally, should HMGB1 purely reflect seizure activity, then one would expect those patients with the most recent seizures to express higher levels of the biomarker. We did not find this to be case in our studies (Supplemental Figure 15). Taken together, these data support a role for HMGB1 in disease pathogenesis and not purely ongoing seizures. With regard to the issue of gliosis, animal data show that the blood changes in HMGB1 did not solely reflect reactive astrogliosis, since the hippocampal level of myo-inositol, a metabolite that mirrors astrocyte activation, was similarly augmented in rats either with or without an increase in blood HMGB1 (Supplemental Figure 12A). Moreover, the level of gliosis assessed in the same rats 7.5 months after SE by postmortem GFAP immunostaining was similar in the hippocampus of rats with epilepsy (showing elevated blood HMGB1) or without epilepsy (with no elevation of blood HMGB1) (Supplemental Figure 12B).

RETRACTED

In order to assess potential therapeutic interventions, our pharmacological study in the electrical SE epilepsy model showed that antiinflammatory drugs targeting the IL1-R1/TLR4 axis significantly (*P* < 0.05) improved the natural history of the disease and prevented elevation of the pathological disulfide isoform in peripheral blood from disease onset. This evidence suggests that blood HMGB1 isoforms may predict therapeutic response to antiinflammatory drugs. Furthermore, since the disulfide HMGB1 seems to be the isoform promoting seizure generation (16), it would seem opportune to develop isoform-specific antagonists that are still lacking (46, 47).

In summary, our results show that the acetylated and reduced isoforms of HMGB1 likely indicate the extent of cell dysfunction/injury early after epileptogenic injuries, while the disulfide HMGB1 isoform may identify patients with a pathologic neuroinflammatory milieu. The current prognostic models for seizure recurrence following a first seizure and for seizure remission following a diagnosis of epilepsy are based on clinical factors including age, seizure type, EEG, and MRI (MESS [ref. 48] and SANAD [ref. 49] models), but lack precision. These models could be much improved by the addition of circulating biomarkers such as HMGB1 and its isoforms.

The data presented in this study strongly support further investigations into the utility of total HMGB1 and its isoforms to act as biomarkers for epileptogenesis and predictors of therapeutic effects of new antiinflammatory agents. Indeed, clinical trial designs for novel therapeutics would greatly benefit from noninvasive biomarkers such as HMGB1 that allow early identification of patients at high risk of developing the disorder and those patients who might preferentially respond to disease-modifying treatments.

RETRACTED

## Methods

### Experimental animals.

Experiments in adult rats and P21 (with P1 defined as the day of birth) rats were carried out at the Mario Negri Institute. Adult (250–300 g) and P21 male Sprague-Dawley rats (Charles River Laboratories) were used. Male pups from 4 independent litters were used and were housed with their dams at constant temperature (23°C) and relative humidity (60%) with a fixed 12-hour light/12-hour dark cycle and free access to food and water until weaning at P21. Older animals were housed 1 per cage.

### Pilocarpine-induced SE in P21 rats.

Lithium chloride (3 meq/kg; Merck Sharp & Dohme) was injected i.p. in P20 rats, 18 hours before the s.c. injection of pilocarpine (60 mg/kg; Sigma-Aldrich) (36–38). Controls were age-matched rats injected with lithium chloride and with an equivalent volume of vehicle (PBS, pH 7.4) instead of pilocarpine. All animals received an injection of 10% sucrose in PBS 2 hours after the onset of SE to improve hydration. SE was not interrupted by any drug administration. SE was visually observed, and its onset time and severity were measured in each rat for 6 hours after pilocarpine injection by 2 independent investigators. The following score was used in each animal: score 1 (general automatisms and exploratory behavior); score 2 (stage 5 seizures, bilateral forelimb clonus with rearing and falling). For each score, we measured the time of appearance of the first symptoms. The onset of SE was determined by time of appearance of at least 2 consecutive stage 5 seizures (<5 minutes apart) that subsequently recurred for the duration of the observation period. Behavioral SE was characterized by continuous bilateral forelimb clonus with rearing and falling (stage 5 of Racine’s scale) (50). These rats were electrode implanted with a depth electrode in the hippocampus and a contralateral surface cortical screw electrode (38) under 1.5% isoﬂurane anesthesia at day 75 after SE for subsequent video-EEG monitoring at 7 months after SE for 2 weeks (24/7) for identifying animals developing or not developing epilepsy (Figure 4). At the end of monitoring, rats were tested for their hippocampal ADT. Animals were electrically stimulated via the recording hippocampal electrode using constant current stimulus (1 msec monopolar square waves, 50 Hz for 2 seconds). Determination of the ADT was done using an ascending stepwise procedure (38, 51, 52). The initial stimulus intensity was 50 μA and was increased by 10 μA up to 100 μA, then by 100 μA up to a maximal value of 400 μA by intervals of 1 minute until 1 AD of at least 10 seconds duration was elicited. Twenty-four hours after AD induction, rats were killed for immunohistochemical analysis of HMGB1 and cell loss. Sham-treated animals (*n* = 7) were vehicle injected (not exposed to SE) and used as controls for blood HMGB1 measurements and histological brain analysis.

RETRACTED

### Electrical SE in adult rats.

Rats were implanted under 1.5% isoﬂurane anesthesia with 2 bipolar Teﬂon-insulated stainless-steel depth electrodes placed bilaterally into the temporal pole of the hippocampus (from bregma: anterioposterior [AP] −4.7 mm; mediolateral [ML] ± 5.0 mm; −5.0 mm below dura) (53). Two screw electrodes were positioned over the nasal sinus and the cerebellum and used as ground and reference electrodes, respectively. Electrodes were connected to a multipin socket and secured to the skull by acrylic dental cement. After surgical procedures, rats were treated locally with Cicatrene powder (neomycin and bacitracin supplemented with glycine, l-cysteine, DL-threonine) and injected with ampicillin (100 mg/kg, s.c.) for 4 days to prevent infections. Rats were allowed to recover from surgery in their home cages for 10 days. Before electrical stimulation, EEG baseline hippocampal activity was recorded in freely moving rats for 24 hours. Then rats were unilaterally stimulated (50 Hz, 400 μA peak-to-peak, 1 ms biphasic square waves in 10-second trains delivered every 11 seconds) in the CA3 region of the ventral hippocampus for 60–90 minutes to induce SE according to a well-established protocol (21, 44). EEG was recorded in each rat every 10-minute epoch for 1 minute in the absence of electrical stimulation, i.e., the stimulus-off period. All rats used for subsequent analysis showed an EEG pattern of uninterrupted bilateral spikes in the hippocampi during the stimulus-off period, starting between the first and the fourth epoch of stimulation onwards. These criteria selected rats developing SE that remitted spontaneously within 24 hours from the initial stimulation, then led to subsequent epilepsy development (21, 44). SE was defined by the appearance of continuous spikes in the γ band with amplitude greater than 2× baseline SD and frequency greater than 5 Hz. Use of the γ band reduces the number of movement artefacts in the EEG recording. The end of SE was set as the time the interspike interval became consistently more than 2 seconds.

No pharmacological intervention was done to stop SE, since no mortality is observed in this model. SE was evaluated by EEG analysis measuring its total duration and the number of spikes during the first 24 hours using the Clampfit 9.0 program (Axon Instruments). Power spectral density (PSD) distribution of 5 frequency bands (δ, 1–4 Hz; τ, 4–8 Hz; α, 8–13 Hz; β, 13–30 Hz; γ, 30–40 Hz) was calculated during 20 hours segmented in temporal windows of 4 hours each. Fast Fourier transforms (FFTs) were computed by 50% overlapping sliding windows (1,024 data points each) with Hanning windowing function. EEG data were normalized by dividing the EEG power density at each frequency by the EEG power density averaged across all frequencies (54).

RETRACTED

### Spontaneous seizure detection following electrical SE.

Rats exposed to electrical SE were continuously video-EEG recorded for detection of spontaneous seizures (24 h/d) from SE induction until 2 spontaneous seizures occurred at least 48 hours apart from SE induction (disease onset; Figure 2). In cross-sectional studies (Figure 1), rats were continuously video-EEG monitored from SE induction until time of sacrifice. All EEG seizures were associated with generalized motor seizures (forelimb clonus with or without rearing and/or falling) (21, 55). After spontaneous seizure onset, video-EEG monitoring was discontinued and resumed at 2 and 4 months after SE to determine spontaneous seizure frequency by continuous EEG monitoring for 2 weeks (24/7) (Figure 3). Spontaneous seizures were discrete EEG ictal episodes lasting on average 60 seconds characterized by high-frequency and high-voltage synchronous spike activity and/or multi-spike complexes (21). EEG was recorded using the TWin EEG Recording System connected with a Comet AS-40 32/8 Amplifier (sampling rate, 400 Hz; high-pass filter, 0.3 Hz; low-pass filter, 70 Hz; sensitivity, 2000 mV/cm; Grass-Telefactor). Digitized EEG data were processed using the TWin record and review software. EEG was visually inspected and quantified by 2 independent operators blinded to the treatments.

### Experimental groups in the electrical SE model.

Three distinct cohorts of rats underwent different procedures for sample collection depending on the analysis to be performed. The first set of rats was transcardially perfused at 3 hours, 6 hours, 24 hours, and 4 days (*n* = 5 rats in each group) after electrical SE onset and used for HMGB1 immunohistochemical analysis (Figure 1A and Supplemental Methods). The second set of rats was killed by decapitation at 3 hours, 6 hours, and 4 days (*n* = 5 rats in each group) after electrical SE, and after rapid transcardial PBS perfusion, was used for measurement of HMGB1 and its isoforms in the hippocampi and in the venous blood collected from the heart atrium (Figure 1B). The third set of rats was used for longitudinal blood withdrawal and for the pharmacological experiment (Figures 2 and 3): electrical SE animals were randomly divided into 2 experimental groups (*n* = 9/each group) treated with vehicle (SE+vehicle) or a combination of antiinflammatory drugs (SE+drug) (Supplemental Figure 5A). In these rats, blood was drawn longitudinally using a chronically implanted jugular catheter at representative times of disease development (Supplemental Figure 5A).

RETRACTED

The procedures for animal anesthesia are reported in the respective methodological sections.

### Drug treatment.

The day before electrode implantation, rats were anesthetized with 1.5% isoﬂurane and surgically prepared with jugular catheters (56) for i.v. injection of drugs. This procedure lasted for about 30 minutes.

We used a combination of 2 different antiinflammatory drugs targeting the IL-1R1/TLR4 pathway, a known contributor to seizure mechanisms (4). Specifically, 1 hour after electrical SE onset, rats were injected with an i.v. bolus of anakinra (10 mg/200 μl sterile saline; Biovitrum AB), which is the human recombinant form of the IL-1R1 antagonist (32), and with BoxA (100 μg/200 μl sterile saline, HMGBiotech), a competitive HMGB1 antagonist (33). A second i.v. injection of both drugs was done 5 hours later, then once daily for a total of 7 days. Rats were also injected i.p. with ifenprodil (20 mg/kg tartrate salt, Sanofi-Aventis), the antagonist of the NR2B-NMDAR (34), once daily for 7 days. The dose of each drug and the treatment schedule were rationally designed based on previous evidence of the drug’s therapeutic effects on neurological deficits, cell loss, and seizures in animal models of acute and chronic degeneration and epilepsy (5, 57). This drug combination was designed, since we know that the mere blockade of the IL-1β/IL-1R1 axis in rats during epileptogenesis is not sufficient to modify disease development (20). We also showed that the IL-1β/IL-1R1 axis blockade does not prevent the TLR4 signaling activation in forebrain (20), which itself contributes to epileptogenesis (15). This set of evidence, therefore, indicates that a combination of drugs targeting both IL-1R1 and TLR4 is required for optimizing the therapeutic response. Ifenprodil was used to block the NR2B-NMDAR, which represents 1 key molecular target mediating the increased excitability and seizures induced by IL-1R1/TLR4 pathway activation (5, 16, 35). This pharmacological experiment was designed to determine whether blood HMGB1 predicts the therapeutic response to antiinflammatory drugs or drugs with different mechanisms of action.

We studied the effect of the combined drugs on the following: (a) levels of total HMGB1 and its isoforms in blood (Figure 2), and (b) the development of spontaneous seizures (Figure 3). In this electrical SE model, around 80% of rats showed an average 5-fold increase in the frequency of spontaneous seizures over 4.5 months from the onset of SE, denoting disease progression (i.e., ratio between the number of seizures at 4.5 months and 2.5 months; Figure 3). Sham-operated animals were implanted with electrodes, but not electrically stimulated (sham, *n* = 9), and were used as vehicle-injected controls for blood HMGB1 analysis.

RETRACTED

### Blood collection in rat epilepsy models.

In the cross-sectional studies done in electrical SE rats (Figure 1B), blood was collected by the heart atrium (before transcardial perfusion) at 3 hours, 6 hours, and 4 days after SE onset; in longitudinal studies (Figure 2 and Figure 4), blood was drawn at representative times of disease development in each model. In electrical SE rats, we collected blood by the jugular catheter in lightly restrained animals (Supplemental Figure 5A); in P21 rats, blood was collected longitudinally from the tail vein in animals under light isoflurane anesthesia placed on a warming pad to avoid hypothermia (Supplemental Figure 5C).

Blood was drawn (~ 500 μl) using a butterfly needle (21 gauge) and collected in microtainer tubes. Plasma was isolated according to standard procedures, aliquoted, and stored at –80°C until assayed. This procedure was carried out within 4 hours of blood withdrawal.

### Brain harvesting in electrical SE model for HMGB1 measurements.

Rats were deeply anesthetized using ketamine (150 mg/kg) and medetomidine (2.0 mg/kg), then rapidly perfused via the ascending aorta with 50 mM ice-cold PBS (pH 7.4) for 1 minute to remove blood from brain vessels. Then rats were decapitated, brains removed, and the ventral hippocampi dissected out at 4°C, immediately frozen on dry ice, and stored at −80°C.

Brain preparation for immunohistochemistry and analysis of cell loss is reported in Supplemental Methods.

### Drug-resistant epilepsy patient study.

A total of 65 patients (37 women and 28 men; mean age, 34.8 years; range, 17–65 years) with drug-resistant epilepsy were admitted to the video-EEG monitoring units of the Walton Centre National Health Service (NHS) Foundation Trust (Liverpool, United Kingdom) (*n* = 15, prospective collection 2010–2013) and Tampere University Hospital (*n* = 50, prospective collection 2004–2007), respectively.

All the patients underwent continuous video-EEG monitoring for electroclinical characterization of their seizures as part of the routine clinical evaluation for possible epilepsy surgery. Ictal scalp recordings were obtained using synchronous digital video and 24-channel standard bipolar EEG. Electrodes were placed according to the International 10–20 system (58) with additional mastoid and anterior cheek electrodes. All patients underwent a diagnostic brain MRI examination on a 1.5 Tesla machine (General Electric Signa HD). Seizures and epileptic syndromes were classified according to the International League Against Epilepsy (ILAE) diagnostic criteria (59).

RETRACTED

AEDs were discontinued during monitoring, and photostimulation/sleep deprivation were utilized under direction of the consulting epileptologist. Seizures were categorized as simple partial seizures (SPSs), complex partial seizures (CPSs), or secondarily generalized tonic-clonic seizures (SGTCSs). The first unequivocally verified localized onset seizure during the video-EEG monitoring was considered as the index seizure. Baseline characteristics of the patients are presented in Supplemental Tables 2 and 4. Healthy volunteers (*n* = 74) without history of seizures served as controls (39 women and 35 men; mean age, 34.1 years; range, 19–66 years). Twenty patients with established (diagnosis more than 12 months prior) well-controlled epilepsy (9:11 symptomatic/idiopathic, 12:8 monotherapy/dual therapy) who had been seizure free for longer than 6 months on AED therapy served as epilepsy controls (12 women and 8 men; mean age, 33 years; range, 18–59 years) (Supplemental Tables 3 and 4).

Blood samples were collected at the beginning of the recording. Blood serum was collected and aliquoted, then stored at –80°C until assayed. This procedure was carried out within 4 hours of blood withdrawal. It has been noted that total HMGB1 levels do not change when blood samples are processed and stored within 4 hours (D.J. Antoine, unpublished observations). Moreover, our laboratory has conducted studies that support this observation, which confirms that HMGB1 redox modifications remain consistent when samples are also processed within 4 hours (D.J. Antoine, unpublished observations). Serum samples were assigned random, linked numerical identifiers by the investigator aliquoting the samples.

### Newly diagnosed epilepsy patient study.

Serum samples were obtained from a randomized trial of AED monotherapy in newly diagnosed epilepsy conducted at the Western Infirmary (60). Participants received monotherapy with levetiracetam, lamotrigine, or topiramate irrespective of epilepsy/seizure type and were followed up prospectively until medication failure (substitution or add-on) or for 3 years, whichever was sooner. The trial primarily focused on drug efficacy and tolerability, collecting information on seizures, adverse effects, and comorbidities. Serum samples were also obtained at random and regular intervals thereafter for the purpose of biomarker analyses. For HMGB1 analysis, only those samples that had been stored continuously at –80°C were used and only from trial participants who had a baseline (randomization) sample and at least 1 further sample obtained during follow-up. This cohort comprised 29 patients (16 male) with a mean age at diagnosis of 29 years (range 17–60). Of these 29 patients, 15 had an initial diagnosis of focal epilepsy, 1 had primary generalized epilepsy, and 13 were unclassified at the time of randomization. Subsequent investigation revealed that 2 individuals (1 focal, 1 unclassified) had NEAD. Of the full cohort of 29 patients, 21 had normal MRIs, 6 had focal abnormalities, and 2 were not exposed to MRI (both NEAD patients had normal MRIs).

RETRACTED

### Assessment of total HMGB1.

Nonidentifiable samples were analyzed by an investigator blinded to the identity of the samples. Total HMGB1 level was determined by commercially available ELISA (Shino-Test Corp.) according to the manufacturer’s guidelines, as described previously (61). In brief, thawed samples were centrifuged at 2000 *g* for 1 minute. The 96-well plate was coated with sample diluent to which 10 μl of sample was added in duplicate. Samples were incubated overnight at 37°C for 20 hours. Plates were washed 5 times in wash buffer (400 μl/well) and air dried. Detection antibody solution (100 μl/well) was added for 2 hours at room temperature. Following the subsequent washing step, substrate solutions were added in equal parts (100 μl/well) and incubated at room temperature protected from light with foil seal for 30 minutes. After incubation, the sample plate was read at 450 nm. Results were fitted to the standard curve.

### Analysis of HMGB1 isoforms by electrospray ionization LC/MS.

Nonidentifiable samples were analyzed by an investigator blinded to the identity of the samples. All chemicals and solvents (iodoacetamide [catalog I1149], DTT [catalog D0632], NEM [catalog 04259], trifluoroacetic acid [TFA; catalog 91707-M]) were of the highest available grade (Sigma-Aldrich). Samples were precleared with 50 μl protein G–Sepharose beads for 1 hour at 4°C. Supernatant HMGB1 was immunoprecipitated with 5 μg rabbit anti-HMGB1 (ab18256; Abcam) for 16 hours at 4°C as previously described (22). Free thiol groups within HMGB1 were alkylated for 90 minutes with 10 mM iodoacetamide at 4°C. Cysteine residues in disulfide bonds were then reduced with 30 mM DTT at 4°C for 1 hour, followed by alkylation of newly exposed thiol groups with 90 mM NEM at 4°C for 10 minutes. Samples were subjected to trypsin (Promega) or GluC (New England Biolabs) digestion according to the manufacturer’s instructions and desalted using ZipTip C18 Pipette Tips (Merck Millipore). Characterization of whole protein molecular weights, acetylated lysine residues, or redox modifications on cysteine residues within HMGB1 were determined by whole protein electrospray ionization or MS-MS as described previously (22, 23) using either an AB Sciex QTRAP 5500 or an AB Sciex TripleTOF 5600 (Sciex Inc.). Peptide analysis was determined using an AB Sciex QTRAP 5500 equipped with a NanoSpray II source by in-line liquid chromatography using a U3000 HPLC System (Dionex, Thermo Fisher UK Ltd.) connected to a 180 μm × 20 mm nanoAcquity UPLC C18 trap column and a 75 μm × 15 cm nanoAcquity UPLC BEH130 C18 column via reducing unions. A gradient from 0.05% TFA (v/v) to 50% ACN/0.08% TFA (v/v) in 40 minutes was applied at a flow rate of 200 nl/min. The ionspray potential was set to 2200–3500 V, the nebulizer gas to 19, and the interface heater to 150°C.

RETRACTED

Unblinding and linkage to the clinical information were performed by a second investigator following completion of the analysis in all cases.

### Statistics.

In each animal experiment, no ad interim analysis was done. Sample size was a priori determined based on previous experience with the respective models; endpoints (outcome measures) and statistical tests were prospectively selected. A simple random allocation was applied to assign a subject to a particular experimental group. All efforts were made to minimize the number of animals used and their suffering according to the 3Rs. Data acquisition and analysis were done blindly.

Statistical analysis was performed by GraphPad Prism 6 (GraphPad Software) for Windows using absolute values. Data are presented as mean ± SEM (*n* = number of individual samples). Dot plots of single values are represented in Figure 5A and in Supplemental Figures 4, 7, and 10. Mann–Whitney *U* test for 2 independent groups and 1-way ANOVA followed by Tukey’s post-hoc test or Kruskal-Wallis followed by Dunn’s post-hoc test for more than 2 independent groups were used for statistical analysis of data. Repeated measures 1-way ANOVA was used to compare HMGB1 levels at different time points of disease development in the same group of rats. The performance of HMGB1 as a biomarker was assessed using nonparametric ROC curves; the AUC was calculated and compared with chance (AUC = 0.5). The performance of the biomarker is considered excellent for AUC values close to 1. The progression index was calculated for each rat as the ratio between the total number of seizures experienced between 4.0 and 4.5 months divided by the total number of seizures from 2.0 to 2.5 months in treatment over the vehicle-injected group. The odds in each experimental group were calculated as the ratio between the number of seizures experienced by rats from 4.0 to 4.5 months and the total number of seizures from 2.0 to 2.5 months. The odds ratio was the ratio between the odds of treatment and the vehicle groups. Differences were considered significant at *P* < 0.05.

RETRACTED

For human data, the presence of HMGB1 isoforms in human sera was unknown; therefore, formal sample size calculation was not undertaken a priori. In addition, a limited number of patients were admitted weekly for inpatient video telemetry; therefore, we utilized convenience sampling in this study, as we could include only those that were available. Statistical analysis was performed using SPSS. Baseline total HMGB1 was compared between 65 patients with drug-resistant epilepsy, 20 patients with well-controlled epilepsy, and 74 healthy controls using 1-way ANOVA followed by Dunn’s test. To test for clinical associations with baseline HMGB1, continuous variables (age, epilepsy duration, seizure frequency, index seizure duration) were tested for association using linear regression, binary variables (MRI, EEG normal/abnormal) using 2-tailed *t* test, and categorical variables (sex, epilepsy type, seizure type, number of AEDs) using 1-way ANOVA. Monthly seizure frequency, index seizure duration, and epilepsy duration showed skewed distribution, and the data were log transformed to achieve normality. Due to the multiple tests undertaken, the false discovery rate was also calculated for each test. To test for association between clinical variables and the presence of the disulfide-HMGB1 isoform, continuous variables were tested for association using the *t* test and categorical variables using χ^2^ or Fisher’s exact test.

### Study approval.

All experimental procedures in animals were conducted in conformity with institutional guidelines in compliance with national (decreto legislativo n.26, gazzetta ufficiale March 4, 2014) and international guidelines and laws (EEC Council Directive 86/609, OJ L 358, 1, December 12, 1987; *Guide for the Care and Use of Laboratory Animals*, US National Research Council, 1996) and were reviewed and approved by the intramural ethical committee.

All patients provided written informed consent prior to inclusion in both clinical studies and to contributing sequential serum samples for biomarker analysis. The study protocols for the drug-resistant patient study were approved by the local ethics and research committees of both sites, North West UK REC–Haydock (Manchester, United Kingdom) (10/H1010/55) and the ethics committee of Tampere University Hospital. The prospective epilepsy study was approved by the West Research Ethics Committee, North Glasgow University (Glasgow, United Kingdom) NHS Trust in August 2003 (ref: 03/74, 1).

RETRACTED

## Author contributions

LEW conducted the United Kingdom study in patients with epilepsy, measured total HMGB1 in blood from patients, and drafted the manuscript. FF conducted the pharmacological study in the electrical SE model in adult rats and the relative histological analysis. TR performed HMGB1 immunohistochemistry and conducted the study in P21 rats. ER, KT, GJS, TT, and LW conducted the kainate study in mice. AJ and LP conducted statistical analysis. TA and JP conducted the Finnish study in patients with epilepsy. MJB and GJS conducted the study in newly diagnosed epilepsy. REJ, BKP, and DJA performed the measurements of HMGB1 isoforms. DJA, GJS, and AGM contributed to study design and manuscript drafting. AV and MP supervised all phases of the project and wrote the final manuscript.

## Supplementary Material

Supplemental data

## Figures and Tables

**Figure 1:** Brain and blood HMGB1 measurements during epileptogenesis evoked by electrical SE in adult rats. (**A**) Representative photomicrographs of hippocampi from control rats (sham) or rats at 3 hours, 6 hours, and 4 days after SE (*n* = 5 each group). Top row shows HMGB1 immunoreactivity in cell nuclei (arrows) or in cytoplasm of glial cells (arrowheads). Immunofluorescence panels show localization of HMGB1 signal (green) in OX-42–positive microglia (red), GFAP-positive astrocytes (red), and EBA-positive endothelial cells (red); colocalization signal is depicted in yellow (merge). White arrows depict cytoplasmic staining. Hoechst-positive nuclei are shown in blue. Rad, stratum radiatum; LMol, stratum lacunosum moleculare. Scale bars: 25 μm (top row); 20 μm (bottom row; immunofluorescence panels). (**B**) Levels of HMGB1 isoforms in brain tissue (hippocampus) and corresponding blood of rats during epileptogenesis. Data are shown as mean ± SEM (*n* = 5 each group). Dot plots are shown in Supplemental Figure 4. *P < 0.05; **P < 0.01, Kruskal-Wallis test (referred to both isoforms in each bar). Blood acetylated and disulfide HMGB1 levels at 4 days are significantly different from corresponding 3-hour and 6-hour levels (*P* < 0.01).

**Figure 2:** Blood HMGB1 levels increase before epilepsy onset in electrical SE–exposed rats and predict therapeutic response to antiinflammatory drugs. Longitudinal analysis of total HMGB1 and levels of acetylated, reduced, and disulfide isoforms in blood plasma at representative time points of disease development in SE-exposed rats receiving treatment (drug) or corresponding vehicle (see key). Treatment included anakinra+BoxA+ifenprodil (SE+drug) (detailed protocol in Methods; Supplemental Figure 5A). Data are shown as mean ± SEM (*n* = 9 rats each group; dot plots are shown in Supplemental Figure 7). Rats are the same as reported in Figure 3. *P < 0.05; **P < 0.01, 1-way ANOVA (referred to both isoforms in each bar, except for prodromal phase, where *P* < 0.01 in SE+drug versus SE+vehicle refers only to reduced HMGB1). The acetylated isoform level in the chronic epilepsy phase (SE+vehicle) was significantly different from corresponding levels at disease onset and prodromal phases (*P* < 0.01, repeated measures 1-way ANOVA). The disulfide isoform (SE+vehicle) level at disease onset and in the chronic epilepsy phase was significantly different from the corresponding level in the prodromal phase (*P* < 0.05 and *P* < 0.01, respectively); the disulfide isoform level in the chronic phase was significantly different from the corresponding level at disease onset (*P* < 0.05, repeated measures 1-way ANOVA).

RETRACTED

**Figure 3:** Antiinflammatory drugs administered during epileptogenesis prevent disease progression in electrical SE–exposed rats. (**A**) Progression index (the ratio between the number of seizures at 4.5 months and at 2.5 months after SE) in vehicle- and drug-treated rats. Value equivalent to 1 defines lack of progression. Data are shown as mean ± SEM (*n* = 9 rats each group). *P < 0.05 versus vehicle, Mann-Whitney *U* test. Raw data are shown in Supplemental Table 1. (**B**) Odds ratio (0.24; *P* = 0.008) indicates that drug-treated rats evaluated at 2.5 months have a 76% reduced risk of developing seizures at 4.5 months versus vehicle-treated rats. Treatment included anakinra+BoxA+ifenprodil (SE+drug) (see Methods; Supplemental Figure 5A). OR, odds ratio.

**Figure 4:** Early prediction of epilepsy development by monitoring blood HMGB1 level in lithium+pilocarpine SE rats. (**A**) Longitudinal analysis of total HMGB1 and acetylated, reduced, and disulfide isoform levels in blood at representative time points of disease development (see key in **A**). Blood was drawn at 23 days (epileptogenic phase prodromal to epilepsy onset), 73 days (encompassing the time of disease onset in 70% of rats), and 7.5 months (chronic epilepsy). Data represent mean ± SEM; *n* = 7 sham; *n* = 5 epileptic (Epi); *n* = 5 nonepileptic (Nonepi) rats. Dot plots are shown in Supplemental Figure 10. **P < 0.01 (refers to both isoforms in each bar); *P* < 0.05, acetylated HMGB1 in epileptic versus sham, Kruskal-Wallis test. Total HMGB1, acetylated and disulfide isoform levels in the chronic phase (Epi) are significantly different versus corresponding levels in prodromal phase (*P* < 0.01, repeated measures 1-way ANOVA). (**B**) Representative immunohistochemical pictures of CA1 stratum radiatum depicting HMGB1 staining in control (sham, *n* = 7) and in SE rats with (Epi, *n* = 5 out of 12) or without (Nonepi, *n* = 5) spontaneous seizures. Rats are the same as reported in **A**. Brains were harvested 7.5 months after SE. Arrows, nuclear staining of HMGB1 in sham and nonepileptic rats; arrowheads, cytoplasmic HMGB1 staining in glia in epileptic rats. Scale bar: 15 μm.

RETRACTED

**Figure 5:** HMGB1 levels in blood of drug-resistant and drug-sensitive epilepsy patients and healthy controls. (**A**) Total HMGB1 levels in healthy controls (1.1 ± 0.07 ng/ml, *n* = 74) and patients with well-controlled epilepsy (1.2 ± 0.15 ng/ml, *n* = 20) or drug-resistant epilepsy (8.7 ± 0.47 ng/ml, *n* = 65; *P* < 0.01). Acetylated HMGB1 was detectable only in patients with drug-resistant epilepsy, and these individuals could be further stratified on the basis of the presence of disulfide HMGB1 (drug-resistant, reduced HMGB1 7.1 ± 0.4 ng/ml, *n* = 41; reduced+disulfide, 11.0 ± 0.9 ng/ml, *n* = 24; *P* < 0.01). Data are presented in each group as individual values as well as the mean ± SEM. **P < 0.01, 1-way ANOVA. (**B**) ROC analysis shows that total HMGB1 discriminates (AUC = 0.99) between patients with drug-resistant seizures and both healthy controls and those with well-controlled seizures.

**Table 2:** Receiver operating characteristic analysis related to Figure 4A

**Table 1:** Receiver operating characteristic analysis related to Figure 2
